RETRACTED

# Multislice Computed Tomography Angiography Imaging Diagnosis of Lower Extremity Arteriosclerosis in Patients with Hypertension and Its Correlation with the Level of High-Sensitivity C-Reactive Protein

**DOI:** 10.1155/2022/1768208

**Published:** 2022-08-31

**Authors:** Jing Huo, Zhongyin Wu, Haijun Jiang, Hong Zhang

**Affiliations:** ^1^Department of General Medicine, Affiliated Hospital of Chengde Medical College, Chengde, 067000 Hebei, China; ^2^Department of Vascular Surgery, Affiliated Hospital of Chengde Medical College, Chengde, 067000 Hebei, China

## Abstract

The aim of this study was to investigate the relationship between multislice computed tomography (CT) angiography (MSCTA) imaging and high-sensitivity C-reactive protein (hs-CRP) in patients with hypertension and lower extremity arteriosclerosis. 68 hypertensive patients with lower extremity arteriosclerosis were selected as the observation group, and 68 healthy volunteers were selected as the control group to compare the differences in hs-CRP. According to the degree of stenosis, the patients were further divided into five grades: no obvious stenosis, mild stenosis, moderate stenosis, severe stenosis, and occlusion. The correlation between the degree of stenosis and the content of hs-CRP was compared. The changes of hs-CRP content before and after treatment were compared, and the difference of images before and after surgical treatment and the difference of hs-CRP expression in patients with occlusion were compared. Compared with the control group, the content of hs-CRP in the observation group was significantly higher (*P* < 0.05), and the degree of stenosis was positively correlated with the content of hs-CRP. After two weeks of treatment, the hs-CRP levels of patients with severe stenosis and occlusion were significantly lower than those before treatment (*P* < 0.01). The level of hs-CRP in patients with occlusion after arterial stent intervention was significantly lower than before, and the images also showed that the blood vessels were significantly expanded. The degree of stenosis in patients with lower extremity arteriosclerosis diagnosed by MSCTA imaging was closely related to the expression of hs-CRP in the patient, and a sustained high concentration of hs-CRP corresponded to a more severe degree of vascular occlusion. In conclusion, the hs-CRP can be used as one of the factors to predict and evaluate the occurrence of cardiovascular and cerebrovascular diseases.

## 1. Introduction

Worldwide, approximately 200 million people suffer from occlusion arteriosclerosis, which can be life-threatening in some cases [1]. Lower extremity arteriosclerosis is the manifestation of occlusion arteriosclerosis in the lower extremities. Occlusion arteriosclerosis is more common in the medium and large arteries at the lower end of the abdominal aorta. Due to atherosclerotic plaque and its internal hemorrhage or plaque rupture, secondary thrombosis leads to gradual lumen stenosis or occlusion, resulting in limb ischemia and other clinical manifestations [2, 3]. With the improvement of social living standards and the aging of the population, the incidence of lower extremity arteriosclerosis occlusion is increasing year by year. The main risk factors of lower extremity arteriosclerosis occlusion disease are hypertension, diabetes, hyperlipidemia, smoking, advanced age, etc. [4]. Studies have found that smoking and diabetes are the most harmful and can increase the incidence of arterial disease by 3 ~ 4 times [5]. The clinical manifestations are intermittent claudication and pain at rest, which can lead to dry gangrene or ulceration in severe cases [6]. Hypertension is one of the risk factors for arteriosclerotic occlusion disease. Although the risk is not as good as diabetes and hyperlipidemia, the number of people suffering from hypertension is large, and it is also a cause that cannot be ignored [7]. Generally speaking, hypertension will cause a relatively large impact on the inner wall of the blood vessel, which will damage the inner wall of the blood vessel after a long time. After the function of the endothelium is damaged, the lipids in the blood are more likely to be deposited on the blood vessel wall, which promotes the occurrence and development of atherosclerosis [8]. On the contrary, the normal diastolic function of the blood vessels with atherosclerosis is weakened, the stiffness of the blood vessel wall increases, and the blood pressure rises again [9].

RETRACTED

Multislice spiral computed tomography (CT) angiography (MSCTA) technology is the application of multislice spiral CT technology in angiography. It can quickly scan a large area without loss of spatial resolution, so that the carotid artery can be better displayed, and the aorta, iliac artery, and femoral artery can also be observed in one scan, effectively using intravascular contrast medium [10]. Because multilayer C can choose thinner layer thickness, the vascular tree of each part can be displayed with higher contrast, which is incomparable with single-layer spiral CT. MSCTA postimage processing techniques include multiplanar reconstruction (MPR), maximum density projection (MIP), volume reconstruction (AR), surface occlusion display (SSD), and simulated inner diameter display (VE) [10, 11]. MSCTA has gradually become an important method for the diagnosis of lower extremity vascular lesions because of its advantages of faster speed, thinner layers, and wider scanning.

High-sensitivity C-reactive protein (hs-CRP) is a nonspecific marker of acute phase systemic inflammation synthesized by the liver. It also specifically refers to C-reactive protein in plasma, which can clinically guide cardiovascular disease, neonatal bacterial infection, and kidney transplantation [12, 13]. Persistent low-level inflammation plays a major role in atherosclerosis, which produces aseptic inflammation due to accumulation of cholesterol and other lipids, resulting in elevated hs-CRP [14]. A large number of studies have shown that high-sensitivity C-reactive protein is mainly located in atherosclerotic plaques and can regulate monocyte aggregation. hs-CRP is a complement activator that coexists with membrane attack complexes in early atherosclerotic lesions, stimulates tissue factor production, and aggregated hs-CRP activates complement. Due to the activation of complement by chronic trace inflammatory factors, lipids are deposited on the vascular wall, and through infiltration and aggregation, vascular damage and atherosclerosis are caused [15]. Studies have found that hs-CRP can chemotactic monocytes at the site of vascular sclerosis, induce monocytes to produce tissue factor, activate complement, induce endothelial cells to produce adhesion factors, impair endothelial function, and accelerate the progression of arteriosclerosis. hs-CRP can also bind to lipoproteins, activate the complement system by the classical pathway, and then generate a large number of terminal complexes, causing vascular endothelial damage [16].

## 2. Methods

### 2.1. Data and Grouping

A total of 68 hypertension patients with lower extremity arteriosclerosis who underwent MSCTA examination in the hospital from January 2020 to January 2021 were selected as the observation group. Clinical manifestations included intermittent claudication, rest pain and/or night pain, pale skin, coolness or numbness, weakness, swelling or muscle atrophy of the affected limb, decreased skin temperature, ischemic cyanosis, gangrene, ulcer, thromboocclusion vasculitis (Buerger) syndrome (+), the pulse of the affected limb femoral artery, popliteal artery, posterior tibial artery, and dorsal foot artery. During the same period, 68 healthy volunteers were selected as the control group for the determination of the content of hs-CRP. This experiment was approved by the ethics committee of the hospital, and all experimental cases obtained the consent of the patients or their families and signed the informed consent.

Inclusive criteria are as follows: (i) hypertensive patients diagnosed as arteriosclerosis of lower limbs by MSCTA examination, (ii) at least 18 years old, and (iii) no history of contrast agent allergy.

RETRACTED

Exclusion criteria are as follows: (i) patients whose lower extremity arteriosclerosis was caused by hyperlipidemia, diabetes, etc.; (ii) patients suffering from arteriosclerosis in other parts of the body and patients suffering from other cardiovascular diseases; (iii) patients suffering from serious body infections; (iv) patients who received kidney transplantation within the past month; and (v) patients who underwent intervention and surgical treatment.

### 2.2. Examination and Treatment

For the treatment of hypertension, oral nifedipine sustained-release tablets II was used twice a day in the morning and evening with a 12-hour interval. For patients with severe claudication, it should take some arterial dilation drugs (cilostazol), antiplatelet drugs (aspirin), or anticoagulant drugs (rivaroxaban) as prescribed by a doctor and prescribe some pain relievers if necessary. Patients with gangrene of limb ulcers required endovascular therapy and surgery. Conventional treatment included ① quitting smoking, which can significantly delay the further aggravation of the disease; ② reasonable arrangement of meals; ③ appropriate exercise to improve ischemia; and ④ attention to foot care to avoid limb injury. All patients were treated with antihypertensive and conventional treatment. No other treatment was performed if there was no obvious stenosis. Arterial dilation, antiplatelet, and anticoagulant drug treatment were performed for mild, moderate, and severe stenosis. Interventional therapy was performed for patients with occlusion, and reexamination should be performed six months after the end of treatment. For patients undergoing interventional therapy, MSCTA was detected, and the images were processed and analyzed using maximum density projection, volume reconstruction, and surface reconstruction techniques and were compared with the lower extremity arterial images of healthy volunteers.

3 mL of fasting venous blood was collected from patients in the observation group in the next morning after admission. The specific protein analyzer was used for inspection, and the content of high-sensitivity C-reactive protein in blood was obtained after analysis. The detection of hs-CRP in healthy volunteers was the same as above.

According to the patient's condition of lower extremity arteriosclerosis, the treatment should be carried out reasonably, and blood collection should be performed to detect the content of hs-CRP in the first and second weeks of drug treatment, conventional treatment, and interventional treatment. After treatment, the content of hs-CRP in patients with each stenosis grade was counted.

RETRACTED

### 2.3. Stenosis Grading Method

The imaging data of MSCTA of 68 patients in the observation group were evaluated by two senior radiologists in a double-blind evaluation of the blood vessels of the lower extremities. The degree of stenosis of blood vessels in CTA-MIP and CTA-VR of the same patient was evaluated, respectively, and CTA-MPR technical analysis could be done if necessary. The lower extremity arteries were divided into 10 segments: lower abdominal aorta, common iliac artery, internal iliac artery, external iliac artery, femoral artery, popliteal artery, tibiofibular trunk, anterior tibial artery, posterior tibial artery, and peroneal artery. Each segment of blood vessels was graded into 5 grades according to the degree of stenosis. The calculation equation of the degree of stenosis was given as follows: degree of stenosis = [(diameter of the normal blood vessel at the proximal end of the stenosis − diameter of the blood vessel at the stenosis)/diameter of the normal blood vessel at the proximal end of the stenosis] × 100%.

Patients with multiple stenosis were classified according to the highest stenosis grade. The patients were grouped according to the grade of stenosis. The specific grades were shown in Table 1.

### 2.4. Data Processing Method

SPSS 23.0 software was used for statistical analysis of the data in this study. All data were expressed as mean ± standard deviation, the counting data are expressed as frequency, the data between observation groups were compared by *t*-test, and the data between multiple groups was compared by one-way analysis of variance. *P* < 0.05 indicated statistical significance.

## 3. Results

### 3.1. Data Statistics and Comparison

As shown in Table 2, the average age of healthy volunteers was 56.23 ± 4.78 years old, and the patients with lower extremity arterial stenosis were 40 males and 28 females, with an average age of 52.13 ± 5.13. There was no significant difference between the patients with lower extremity arteriosclerosis and the healthy persons in the clinical basic data (*P* > 0.05). In addition, according to the judgment of the doctor and the evaluation of the stenosis grade, the statistics of the number of volunteers with each stenosis grade were shown in Figure 1. 19 patients had no significant stenosis, 18 had mild stenosis, 15 had moderate stenosis, 9 had severe stenosis, and 7 had occlusion (Figure 1).

### 3.2. Comparison of the Content of hs-CRP

As shown in Figure 2, the content of hs-CRP in the plasma of patients with lower extremity arteriosclerosis was 1.26 ± 0.21 mg/L and that of healthy volunteers was 15.13 ± 4.42 mg/L. After comparison, it was found that there was a significant difference in the content of hs-CRP between the two groups (*P* < 0.01). This also showed that the plasma hs-CRP of patients with lower extremity arteriosclerosis was significantly higher than that of healthy volunteers.

RETRACTED

### 3.3. Analysis of hs-CRP Content in Each Stenosis Group

The patients with lower extremity arterial stenosis in the observation group were regrouped according to the degree of stenosis, and the average levels of hs-CRP in each group were counted, as shown in Figure 3. Starting from the moderate stenosis group to severe stenosis group, each group had a significant difference compared with the previous group (*P* < 0.05). There was no significant difference in complete vascular occlusion compared to the severe stenosis group. This also showed that with the increase in the degree of stenosis, the patient's plasma hs-CRP also increased.

### 3.4. Comparison of hs-CRP Content after Treatment

As shown in Figure 4, patients with no obvious stenosis and mild stenosis had no significant change after comprehensive treatment compared with before treatment, and there was no significant difference after comparison (*P* < 0.05). Compared with before treatment, the content of hs-CRP in patients with moderate stenosis was significantly lower after two weeks of treatment, and the difference was statistically significant (*P* < 0.05).

### 3.5. MSCTA Imaging and hs-CRP Analysis before and after Interventional Therapy

A patient with right femoral artery occlusion was diagnosed with MSCTA on admission and analyzed using maximum density projection and boneless volume reconstruction techniques. Afterwards, under the doctor's suggestion, he underwent femoral artery stent implantation, and he came to the hospital for reexamination and diagnosis. The patient's hs-CRP concentration at the first examination was 15.17 mg/L, as shown in the images after MSCTA imaging (Figures 5(c) and 5(d)). Compared with the blood vessels of healthy volunteers (Figures 5(a) and 5(b)), the patient's right femoral artery was significantly occlusion, with collateral circulation, the left femoral artery was narrowed and severely calcified, and the left tibial anterior and posterior tibial arteries were tiny. Six months after the right side received femoral artery stent implantation, the hs-crp concentration was 9.51 mg/L, which was significantly lower than that before treatment. After the consultation, it was found that the recovery state was good, and further reexamination, CT plain scan (Figure 5(e)) found that the stent was unobstructed, and no stenosis and thrombosis were found. The implanted vascular stent can be clearly seen in the CTA surface reconstruction (Figure 5(f)), the boneless volume reconstruction (Figure 5(g)), and the maximum density projection (Figure 5(h)).

RETRACTED

## 4. Discussion

hs-CRP is an effective and sensitive marker of inflammation in vivo, which marks the acute phase of inflammation and can predict the occurrence of cardiovascular and cerebrovascular events. The process of atherosclerotic lesions is closely related to the inflammatory response caused by continuous and repeated damage of blood vessels. hs-CRP can activate phagocytes, activate complement, make vascular endothelial cells dysfunctional, promote foam cell formation, inhibit the survival and differentiation of endothelial progenitor cells, activate the intima of atherosclerosis, and further lead to the occurrence of atherosclerosis [17]. The results of this work found that patients with higher arterial stenosis had higher plasma hs-CRP, which to some extent indicated that patients with lower extremity arteriosclerosis caused by hypertension already had a certain inflammatory response. Therefore, in addition to MSCTA, hs-CRP can also be used as a reference index for the degree of disease. In a study on the association between hs-CRP and clinical outcomes in patients with intermittent claudication in the past decade, it was found that elevated hs-CRP levels were significantly associated with cardiovascular-related and cancer-related deaths in patients with intermittent claudication [18]. In the study of psoriasis and cardiovascular disease risk, it was found that patients with psoriasis had a higher risk of subclinical atherosclerosis. hs-CRP is a useful marker of cardiovascular disease risk, and anti-inflammatory drugs not only play a key role in the treatment of psoriasis but also reduce cardiovascular risk by reducing levels of inflammatory markers including hs-CRP risk of disease [19]. In the study of the relationship between ultrasound and hs-CRP and carotid stenosis, it was found that high hs-CRP and the degree of carotid stenosis were closely related [20].

Digital subtraction angiography (DSA) has always been the gold standard for diagnosing lower extremity arteriosclerosis occlusion, but its disadvantage is trauma examination [21]. However, with the development and improvement of MSCTA, it has become the mainstream way of examining arterial blood vessels. In addition to its advantages of convenience, noninvasiveness, and high patient acceptance, MSCTA can more intuitively display the length of arterial vessels, the degree of stenosis, collateral circulation, and perivascular tissue. MSCTA has many image processing methods, and different processing techniques can be selected according to needs, which can provide a variety of rich image data for clinical practice [22]. In this work, the stenosis of lower extremity arteries can be clearly observed and classified according to the degree of stenosis by selecting maximum density projection, solvent reconstruction, and multiplanar reconstruction technology after MSCTA scanning. A study using MSCTA and DSA techniques to differentiate the internal iliac artery branch angiography in patients with pelvic tumors found that MSCTA has a great advantage over DSA in the evaluation of the branch vessels at the end of the internal iliac artery [23].

RETRACTED

Since MSCTA can well analyze the degree of stenosis of blood vessels in patients through various imaging systems and hs-CRP is an important marker of vascular stenosis, there must be a certain correlation between the two. This experiment also found that the higher the stenosis degree, the higher the hs-CRP level of the patients, and the hs-CRP level of the patients with a high degree of stenosis was significantly different from that of the patients with a lower degree of stenosis (*P* < 0.05). In addition, this work also studied the hs-CRP level of patients after corresponding treatment of arteriosclerosis. The results showed that after treatment, the level of hs-CRP in patients with severe stenosis and occlusion was significantly reduced after two weeks of treatment (*P* < 0.01). A six-month follow-up visit to a patient with vascular occlusion treated with interventional stents also found that the occlusion blood vessels of the lower extremities were completely unblocked, and the level of hs-CRP in the body was significantly lower than before treatment. All the above experiments showed that the degree of vascular stenosis determined by MSCTA was closely related to the level of hs-CRP.

## 5. Conclusion

MSCTA imaging can clearly observe the degree of stenosis of lower extremity arteries, and it is also found that the level of hs-CRP in patients with hypertension is closely related to the degree of stenosis of lower extremity arteriosclerosis. Patients with severe vascular stenosis tend to have higher levels of hs-CRP in plasma. After treatment, patients' lower extremity vascular stenosis is reduced, and hs-CRP levels are also reduced. The disadvantage of this experiment is that there are too few experimental samples, which cannot more accurately reflect the relationship between MSCTA imaging and hs-CRP. In addition, considering that the treatment method is different for each patient, there was no significant difference in the hs-CRP level between mild and moderate patients before and after treatment. In follow-up studies, more experimental samples should be sought, especially to include more patients with severe stenosis and occlusion, and to develop better treatment modalities for classification.

RETRACTED

## Figures and Tables

**Figure 1:** Distribution of the number of patients by degree of stenosis.

**Figure 2:** Comparison of the concentration of hs-CRP in the plasma of the control group and the observation group. ^∗^Compared with the control group, *P* < 0.01.

**Figure 3:** Comparison of concentrations of hs-CRP in each stenosis group. ^∗^Compared withthe insignificant stenosis group, *P* < 0.05; ^#^compared with the mild stenosis group, *P* < 0.05; ^^^compared with the moderate stenosis group, *P* < 0.05.

**Figure 4:** Expression of hs-CRP in each stenosis group after comprehensive treatment. (a–e) The expression levels of hs-CRP before treatment and after one week and two weeks of treatment in each group with no obvious stenosis, mild stenosis, moderate stenosis, severe stenosis, and occlusion, respectively. ^∗^Compared with that before treatment, *P* < 0.05; ^#^compared with that before treatment, *P* < 0.01.

**Figure 5:** Comparison of MSCTA imaging processing before and after stent implantation in patients with lower extremity arterial occlusion. The marked part in red indicated the narrow part of the lower limb artery. (a, b) The imaging results of blood vessels of healthy volunteers. (c, d) The imaging results of the blood vessels of patients. (e) The CT plain scan results. (f) The CTA surface reconstructed image. (g) The image after boneless volume reconstruction. (h) The image constructed by the maximum density projection.

**Table 1:** Criteria for stenosis grading.

Grade	Degree of stenosis
Grade 1	No obvious stenosis
Grade 2	Mild stenosis (<50%)
Grade 3	Moderate stenosis (50%-70%)
Grade 4	Severe stenosis (71-99%)
Grade 5	Occlusion

**Table 2:** Comparison of clinical data.

Group	Cases	Gender		Age (years old)
		Males	Females	
Control group	68	37	31	56.23 ± 4.78
Observation group	68	40	28	52.13 ± 5.13

## Data Availability

The data used to support the findings of this study are available from the corresponding author upon request.
